The article "Research on the Communication Strategy of History and Culture in Shaanxi Based on BP Neural Network Model" was published in 2022. Journal: Comput Intell Neurosci.

# Research on the Communication Strategy of History and Culture in Shaanxi Based on BP Neural Network Model

**DOI:** 10.1155/2022/8965622

**Published:** 2022-01-24

**Authors:** Dan Xie, Chao Yin

**Affiliations:** ^1^General Department, Xi'an Traffic Engineering Institute, Xi'an 710300, Shaanxi, China; ^2^University of Technology MARA, Shah Anam, Selangor 40450, Malaysia; ^3^School of History and Culture, Shaanxi Normal University, Xi'an 710000, Shaanxi, China; ^4^Xi'an Tie Yi Middle School, Xi'an 710000, Shaanxi, China

## Abstract

Shaanxi is one of China's most important cradles of civilization. The main vein of Chinese culture is rich history and culture, and brilliant red culture embodies the essence of socialist core values. It is still relatively weak to deeply analyze the related research of Shaanxi Province's cultural province construction on the basis of studying the achievements of cultural development in foreign countries and China and combining with the reality of Shaanxi Province. In this paper, a BPNN (BP neural network) model is selected to study the comprehensive evaluation of tourism competitiveness of smart tourism cities, and the software is used to realize the simulation of the comprehensive evaluation system of tourism competitiveness of smart tourism cities, which more comprehensively and objectively reflects the level of comprehensive competitiveness of each city. It is believed that there are some problems in Shaanxi regional cultural communication, such as insufficient exploration of content resources, insufficient communication channels, and low audience awareness, hoping to provide ideas and reference for further exploring the promotion of cultural communication power.

## 1. Introduction

Shaanxi is recognized as a province with rich cultural resources and is vigorously building Shaanxi as a province with rich historical culture, splendid revolutionary culture, distinctive folk culture, and modern culture with certain strength. How to develop Shaanxi's cultural undertakings with the help of rich cultural resources and develop a culturally rich province into a culturally strong province has become the direction of the joint efforts of provincial party committees and governments [1]. Although Shaanxi has made great achievements in the development of cultural undertakings and cultural industries in recent years, it is not commensurate with the requirements of being a big cultural province and building a strong cultural province. Compared with developed provinces, there is still a big gap, and the construction of a strong cultural province still faces some problems and difficulties [2, 3]. This is also the background of this topic.

The article "Research on the Communication Strategy of History and Culture in Shaanxi Based on BP Neural Network Model" was published in 2022. Journal: Comput Intell Neurosci.

Many cultural communication professionals began to actively study the internal relationship between the Internet and cultural communication content in the era of mobile Internet to better understand how to spread cultural content through the Internet. Cultural construction is an important aspect of socialist construction and a crucial component of the Chinese style socialist theoretical system. The classification and planning of historical and cultural cities, as well as the attention paid to implementation after the planning of famous city protection, are clearly inadequate. Protection planning should not be a one-size-fits-all approach [4, 5]. Protection planning should be evaluated in light of changes in implementation as protection work progresses, and this should be used as the basis for planning adjustments [6]. To enrich Shaanxi's cultural construction, it is critical to study the construction of Shaanxi Province as a strong cultural province. This paper examines the problems and reasons for the construction of a strong culture in Shaanxi Province, as well as the countermeasures and recommendations for the construction of a strong culture in Shaanxi Province, which is of reference value to the country's and other provinces' cultural construction.

Beginning with the scientific definition of culture, this paper examines the current state of Shaanxi's cultural province construction, highlighting the accomplishments and benefits of Shaanxi's cultural construction, and identifying the major issues that exist in Shaanxi's cultural construction. A transportation mode selection model based on the BPNN (back propagation neural network) algorithm is established after comprehensively considering the attribute variables and activity patterns of travelers, with a focus on the historical block, a special block. Using the protection of ancient cities as an example, it has been demonstrated that the BPNN evaluation model of the entire process of historic city protection planning can be used for historic city protection evaluation.

## 2. Related Work

The early research mainly focused on the background of cross-cultural generation, while the current research has already involved many disciplines of humanities and social sciences [7, 8]. Yang et al. [9] propose that some information is hidden in the context when people communicate with each other, and there are different levels of communication contexts among countries and ethnic groups. Countries such as Britain and the United States belong to the low-context society, while countries such as Japan and South Korea belong to the high-context society. By analyzing the current situation of foreign language education in China, Liu and Hu [10] pointed out that foreign language teaching in China attaches importance to language knowledge and language skills but neglects the cultivation of cultural factors, so that Chinese college students lack intercultural communication skills. Based on this, Hou [11] proposes to build a brand-new college English-teaching model based on intercultural communication. Wu and Ma et al. [12, 13] propose that to achieve effective communication across the gap of nationality, race, nationality, language, and culture, it is necessary to search for and think about the multidimensional interaction between self, people and society, people and culture, people and media, so as to find out the possible path of cross-cultural communication. Zhan [14] discusses smart tourism in depth and thinks that smart cities should have six dimensions: smart economy, smart environment, smart transportation space, smart people, smart families, and smart government. Through data analysis, it is found that innovation ability, attention to urban environmental quality, administrative management, and education level play an important role in the utilization of information technology and the intelligence of cities [15, 16].

The article "Research on the Communication Strategy of History and Culture in Shaanxi Based on BP Neural Network Model" was published in 2022. Journal: Comput Intell Neurosci.

The characteristics of artificial neural networks in terms of information processing are unique. It has been used successfully in a variety of fields. It has strong nonlinear mapping capabilities, as well as self-adaptation, self-learning, fault tolerance, and parallel processing capabilities. Neural networks have properties that make them ideal for studying chaotic sequence prediction. The use of neural networks [17] in multivariable time-series prediction and multivalue prediction has been studied in literature [18, 19], and Lu et al. [20] discuss the modeling mechanism and multivalue prediction of this method, as well as its application in stock price prediction. Tang and Yu [21] discuss the establishment mechanism of a time-series prediction model based on neural networks and then propose an adaptive time-series modeling and prediction by combining the time-difference method with BPNN. Sun and Lei [22] developed a radial basis function neural network model using cluster analysis, tested it using financial time series, and compared it to the radial basis function neural network model. Yuan et al. [23] established a time-delayed BPNN model and used the Bayesian regularization method to improve BPNN's generalization ability. Furthermore, many researchers used the search algorithm in optimization to improve the common BP learning method's convergence speed and network prediction performance.

## 3. Research Method

### 3.1. Communication Design of Shaanxi Regional History and Culture

The goal of Shaanxi Province as a strong cultural province is an indispensable part of the construction of “western province”. Attaching great importance to cultural construction ideologically is an important prerequisite for building a strong cultural province. Shaanxi talents will have more sense of belonging and existence. Cultural construction is an important symbol of Shaanxi's comprehensive strength. A country pays attention to comprehensive national strength, and a province also pays attention to comprehensive labor saving, including not only material strength such as economic strength, scientific and technological strength, but also spiritual strength such as culture.

The article "Research on the Communication Strategy of History and Culture in Shaanxi Based on BP Neural Network Model" was published in 2022. Journal: Comput Intell Neurosci.

Culture, as a special component of comprehensive strength, is based on and backed by developed economy. Building a moderately prosperous society, to achieve the goal of building a culturally powerful province in the west also requires firm belief and guidance. Cultural construction provides intellectual support for the construction of a strong western province. China's modernization process, to a great extent, depends on the improvement of national quality and the development of human resources. Shaanxi should be highly aware of the importance of cultural construction ideologically, make full use of the advantages of efficient resources, train outstanding and high-quality talents, and provide backup forces for the construction of Shaanxi's strong cultural province.

As a kind of “soft power”, culture is increasingly becoming an important factor of regional competitiveness and an important aspect of a region's comprehensive strength. Cultural background, cultural environment and atmosphere, and scientific and cultural quality of workers are increasingly becoming the important foundation and guarantee of economic development. The complex relationship between culture and economy is becoming more and more important. Therefore, the significance of cultural revival is not limited to simple economic development.

Thousands of years have passed since many cultural relics, historic sites, and cultural sites in historical and cultural cities were destroyed and rebuilt. They have remained tourist attractions for the time being, due to the cultural continuity and inheritance [24]. Aside from the continuation and inheritance of culture, the cultural sustainable development of famous historical and cultural cities is also very important for the innovation and development of culture, and it is an important index to measure the continuation of “context” of famous historical and cultural cities as well as the development of culture over time. It is a critical ally in the development of cultural tourism. Tourists are drawn to cultural relics and historic sites in well-known historical cities because they are diverse, have a long history, have a high taste, are valuable, and have a high ornamental value. At the same time, the material carriers of culture are the preservation of cultural relics and historic sites in well-known historical and cultural cities, the preservation of ancient architectural styles, and the preservation of cultural landscapes. The cultural evaluation index system of historical and cultural cities includes five major factors, which constitute an index system composed of three levels: target level, factor level, and index factor level, as shown in Figure 1.

The article "Research on the Communication Strategy of History and Culture in Shaanxi Based on BP Neural Network Model" was published in 2022. Journal: Comput Intell Neurosci.

The cultural industry in Shaanxi has more potential for economic growth. Shaanxi takes cultural tourism as a breaking point because of its diverse and colorful cultural resources, and labor drives many economic growth points throughout the industrial chain, including the cultural leisure industry, book publishing industry, and advertising exhibition industry. Culture is, at its core, a creative endeavor. Through the integration of various forms of cultural resources, various cultural products and services with fresh vitality can be continuously produced with the continuous input of creativity.

In the field investigation, the vast majority of tourists are in a positive and high emotional state, and a small number of tourists are mixed with negative emotions. In the specific tourism situation, this paper only selects tourists' positive tourism emotions as the focus of this paper. On the whole, the higher the tourists' positive tourism emotion, the stronger the tourists' sense of experience and identity to the tourist destination, and the greater the tourists' satisfaction. The structural model is shown in Figure 2.

Tourist satisfaction plays a part of intermediary role between positive tourism emotion and behavioral intention. As a senior creature, people's tourism emotion is complex in the process of tourism. The level of tourism emotion depends on tourists' experience and recognition of the tourism world, and its influence is far-reaching and extensive. On one hand, positive tourism emotion affects tourists' satisfaction with tourist destinations, on the other hand, it also has a direct effect on their behavior intention, but at the same time, tourists' positive tourism emotion also plays a role in behavior intention through overall satisfaction.

It is worth noting that while tourists' positive tourism emotion has a strong influence on behavior intention, the impact of positive tourism emotion on behavior intention is weakened when tourists' satisfaction factors are taken into account. As a result, the most important aspect of tourist destination management is to pay attention to tourist satisfaction. Xi'an tourists appreciate the ancient capital's incomparable charm because of its unique tourism resources and beautiful natural and cultural environment. As a result, Xi'an tourists' tourism emotion and satisfaction with tourism resources and culture, tourism environment, and facilities are related in the travel process, and there is a positive correlation. There is, however, no link between tourism emotion and tourism expectations, tourism service, or tourism price. The causal relationship between them cannot be determined using correlation analysis. The next step of regression analysis is required to investigate the relationship between tourists' tourism emotions and tourism resources and culture, tourism environment and facilities, and overall satisfaction.

The article "Research on the Communication Strategy of History and Culture in Shaanxi Based on BP Neural Network Model" was published in 2022. Journal: Comput Intell Neurosci.

### 3.2. BPNN Model Design

#### 3.2.1. BPNN Structure

BPNN algorithm is a training algorithm based on the principle of error back propagation. It takes the minimum error mean square as the criterion and uses nonlinear differentiable function for weight training. BPNN is a multilayer forward anger network, which is composed of IL (Input layer), HL (hidden layer), and OL (Output layer). Usually, the number of layers of neural network does not include IL.  Figure 3 is the BPNN structure diagram.

The HL transfer function of BPNN adopts the nonlinear function of continuously differentiable, usually Sigmoid function, while the transfer function of OL can adopt linear function or Sigmoid function, depending on the distribution range of OL vector.

Basic steps of algorithm: set the initial value of each weight or threshold: *w*_*ji*_(0), *θ*_*j*_(0) is a small random number.

Provide training samples: input vector *X*_*k*_, *k*=1,2,…, *P*; Expected output *d*_*k*_, *k*=1,2,…, *P*;

Calculate the actual output of the network and the state of HL unit:

(1) $$\begin{array}{c} o_{kj}=f_{j}\left(\sum_{i}w_{ji}o_{ki}-\theta_{j}\right). \end{array}$$

Training error:

(2) $$\begin{array}{c} \delta_{kj}=o_{kj}\left(1-o_{kj}\right)\left(t_{kj}-o_{kj}\right),\\ \delta_{kj}=o_{kj}\left(1-o_{kj}\right)\sum_{m}o_{km}w_{mj}. \end{array}$$

Corrected weights and thresholds:

(3) $$\begin{array}{c} w_{ji}\left(t+1\right)=w_{ji}\left(t\right)+\eta \delta_{j}o_{ki}+\alpha \left[w_{ji}\left(t\right)-w_{ji}\left(t-1\right)\right],\\ \theta_{j}\left(t+1\right)=\theta_{j}\left(t\right)+\eta \delta_{j}+\alpha \left[\theta_{j}\left(t\right)-\theta_{j}\left(t-1\right)\right]. \end{array}$$

When *k* goes through 1 to *P*, judge whether the index meets the accuracy requirement.

The article "Research on the Communication Strategy of History and Culture in Shaanxi Based on BP Neural Network Model" was published in 2022. Journal: Comput Intell Neurosci.

#### 3.2.2. Establishment of the BPNN Evaluation Model

To meet the requirements of training error and prediction error, BPNN model training must include a series of constant comparisons between expected value and neural network output value, as well as repeated training and simulation operations. The comprehensive evaluation value of the implementation evaluation of historic city protection planning is obtained using the expert scoring method and is used as the expected value of BPNN model training samples.

The training samples come from 100 randomly generated sample evaluation values. According to the scores, the famous cities are evaluated and divided into five grades: (90–100) as good, (80–89) as good, (70–79) as good, (60–69) as fair and below 60 points as poor. The formula is as follows:

(4) $$\begin{array}{c} P=\sum C_{i}\times W_{i}, \end{array}$$

where *P* is the comprehensive evaluation value for the protection planning of historic cities, *C*_*i*_ is the single score of evaluation index, and *W*_*i*_ is the weight of evaluation index.

#### 3.2.3. Determination of the Number of HL Nodes

In the process of BPNN training, the weights and thresholds change randomly and change with the training times. The number of HL layers and the number of nodes in each layer will directly affect the training results. By setting the number of HL nodes, the training accuracy will be improved, and the error will be reduced. After debugging for many times, the number of HL nodes that reach the required accuracy and error is finally selected, and this number of HL nodes is the final required number of nodes.

There are many ways to determine the number of HL nodes, which are determined by empirical formula in this paper.

(5) $$\begin{array}{c} m=\sqrt{n+I}+a, \end{array}$$

where *n* is the number of IL nodes, *I* is the number of OL nodes, and *a* is a constant from 1 to 10, so it is determined that the number of HL nodes is 13.

Each index has its own dimension. In the process of calculation, for the factors with different equivalent levels, dimensionless measures should be taken to make each factor in the same equivalent level. In this case, to make the input factors dimensionless, the actual travel time should be divided by 10 as the input of travel time, and the other seven factors should be converted into smaller values by stages, so as to avoid unnecessary errors caused by large data gaps and improve the training speed and accuracy.

#### 3.2.4. Training Strategy

The sample data are usually divided into two parts when training the network: one part is used for training, and the other part is used to test the training effect. As BPNN is trained using the gradient descent method, the training set's error will decrease monotonically, while the average error on the test sample set will always be higher than the training sets, which will not decrease monotonically. The big trend is that after reaching a certain training level, the error on the training set decreases first, then increases again. As a result, rather than continuing to train until the error of the test set reaches the minimum point, the network usually stops training when the error of the test set reaches the minimum point.

The article "Research on the Communication Strategy of History and Culture in Shaanxi Based on BP Neural Network Model" was published in 2022. Journal: Comput Intell Neurosci.

## 4. Results Analysis and Discussion

### 4.1. Learning and Training Analysis of the BPNN Method

Shaanxi has a splendid red culture, in which the influence of Yan'an spirit radiates all over the country. Until now, the land of Sanqin has a large number of red cultural resources, including both material cultural resources and historical and cultural heritages, such as revolutionary documents, memorial sites, literary works, cultural relics, revolutionary war sites, and so on. In Shaanxi regional culture, there are many cultural resources rich in popular entertainment and expressive force, particularly some folk arts that are more suitable for media communication. These are priceless gems that must be thoroughly explored and exploited, and brands with distinct label value must be created to ensure strong and effective communication. Furthermore, the development of high-quality content in Shaanxi regional culture must be accelerated. There are some issues right now, such as a low level of innovation transformation, a lack of second creation, and a shallow interpretation.

In traffic mode division, the whole process of BPNN is divided into three steps. First, a suitable neural network must be established. Second, the network should be trained according to the existing input and output data to make the accuracy and error of the network as small as possible. Finally, the output prediction of other input data should be made according to the trained network. Train the network according to the nonlinear function, and get the output of the nonlinear function predicted by the trained network (Figure 4).

It can be seen from Figure 4 that on the basis of training, the remaining 15 pieces of data are used for prediction, and the predicted data basically accord with the expected data, which shows that BPNN algorithm has certain practicability in the research field of transportation mode selection.

Shaanxi's cultural market access conditions are constantly relaxed, but the cultural market order needs to be further standardized. A good cultural market environment is the foundation for the healthy development of the cultural industry. At present, the situation of fragmented, multihead management and fragmented cultural market in Shaanxi exists to a certain extent, which not only increases the difficulty of organizing capital operation but also causes waste and idleness of cultural resources. Cultural development is low and immature, and cultural products lack a standardized market trading environment and have not really formed a perfect market mechanism.

The article "Research on the Communication Strategy of History and Culture in Shaanxi Based on BP Neural Network Model" was published in 2022. Journal: Comput Intell Neurosci.

The above case proves that the BPNN algorithm is practical in the research field of transportation mode selection. The traffic sharing rates of Xi'an, Hanzhong, Luoyang and Baoji in Figure 1 are verified by BPNN method (Figures 5–7).

The verification results show that the predicted data of the traffic mode division model based on BPNN algorithm are basically consistent with the actual survey data.

The rich forms and contents of Shaanxi regional culture necessitate rich communication platforms or channels for all-around communication. In today's world, new media, in addition to traditional media, is a must-have communication channel. It is the audience's cultural communication's arrival terminal, so the effect of cultural communication power will eventually be reflected in the audience as the terminal. The investigation of the effect is primarily based on two levels of cultural awareness and recognition. It is necessary to divide the audience into groups, such as those who live in the province and those who live outside of it. Their understanding of Shaanxi regional culture differs, allowing them to communicate more effectively.

The cultural service system is sound. Public cultural facilities are scientifically planned, rationally laid out, and coordinated between urban and rural areas. Large and medium-sized cities have a number of modern symbolic cultural and entertainment facilities with high level, high standard, and unique style. Comprehensive cultural facilities and places for cultural activities at the grass-roots level are fully functional and basically can meet the needs of the masses to carry out regular cultural activities. The cultural service network is sound, with complete functions, wide coverage, and high service capacity and level.

At present, the dissemination of Shaanxi regional culture is not accurate enough in audience segmentation, which leads to the loss of communication effect. Different audiences have uneven awareness of regional culture, and thus have different recognition of culture. In addition, the content, methods, channels, and skills of cultural communication all have an impact on the final communication effect, and these contents should be based on the accurate research of the audience.

The article "Research on the Communication Strategy of History and Culture in Shaanxi Based on BP Neural Network Model" was published in 2022. Journal: Comput Intell Neurosci.

### 4.2. Evaluation and Analysis of Shaanxi Regional Historical and Cultural Tourism

The research on the tourism competitiveness of smart tourism cities is a hot issue in the current tourism field. Under the development trend of modern tourism with the theme of science and technology and competition, the smart tourism city complex as a tourist destination has a comparative advantage with other smart tourism cities in the competition of tourism elements under the comprehensive action of tourism economic development, scientific and technological innovation, tourism resources, environmental support, geographical location, and other factors.

The tourism competitiveness of smart tourism cities is embodied in five aspects: economic development, scientific and technological innovation, potential competitiveness, environmental support, and development guarantee of smart tourism cities.

According to the established BPNN, relevant training comparison values can be obtained (as shown in Figure 8).

Figure 8 shows that the expected output value is very close to the value of neural network training output value. In other words, the BPNN model can accurately determine the general situation of tourism competitiveness of smart tourism cities according to various evaluation indexes. Therefore, the training of network model is over, and the evaluation model of tourism competitiveness of smart tourism cities based on BPNN has been constructed. When evaluating the tourism competitiveness of other smart tourism cities, only need to enter the normalized data of the evaluation sample index, and the required evaluation conclusion can be obtained.

Based on the results of BPNN evaluation on the competitiveness of smart tourism cities because the competitiveness of each city is different, by comparing other sample cities with those in an advantageous state, smart tourism cities can have an objective understanding of their own level of smart construction and the competitiveness of other cities, identify the gap and take corresponding measures to improve their competitiveness.

After BPNN training, the trained BPNN model is used for testing, and the index data of Xi'an and Shangluo test samples are input into the model, and the output results shown in Figure 9 are obtained.

The error of the test samples is close to the error of the training samples through the trained neural network, and it is assumed that the established network model can effectively approach the training samples based on the test samples in Figure 9. The relative and absolute error values of training and test samples in the BPNN model are also within acceptable bounds. As a result, the BPNN-based evaluation model of smart tourism city competitiveness developed in this paper is effective, and the directly trained neural network can be used to evaluate the competitiveness of other smart tourism cities.

The article "Research on the Communication Strategy of History and Culture in Shaanxi Based on BP Neural Network Model" was published in 2022. Journal: Comput Intell Neurosci.

Through the training results of BPNN, the evaluation results of 10 smart tourism city samples are compared and ranked, and the final competitiveness ranking is shown in Figure 10.

The core of culture is certain values and their concrete norms. Shaanxi is rich in cultural resources, but its influence is limited due to insufficient understanding and development. At the important stage of the transition period, it is necessary to fully understand and explore the spiritual education value of Shaanxi's red cultural resources with Yan'an spirit and patriotism as the main connotation, so as to urge people to reflect on the spiritual emptiness and belief confusion that are prevalent now, draw positive energy from the values, outlook on life and spirit of life of revolutionary ancestors, establish correct value goals and value pursuits, shape social psychology of self-respect and self-improvement, and stimulate initiative and creativity.

Shaanxi is rich in science, education, and culture resources, and it is a big province of science and education, which provides intellectual support and powerful guarantee for the modernization of culture in terms of technology and manpower. The development of culture in the new period cannot be separated from scientific and technological innovation, such as animation industry, film, and television production industry, creative advertising industry and so on, which have highly accumulated scientific and technological content. Give full play to the advantages of Shaanxi education and the strength of science and technology, promote the integrated development of enterprises in Industry-University-Research, realize the linkage between cultural industry capital and intellectual capital, and innovate and develop culture with high technology.

Culture and science and technology are the areas that need innovation most. If you plug in the wings of culture and technology, it will accelerate the transformation of culture and science and technology into real productive forces and maximize the cultural value. Shaanxi has both. As long as attach great importance to and develop reasonably, the resources of science and education will certainly promote the prosperity and development of Shaanxi culture.

## 5. Conclusion

At this new historical juncture, we must deeply comprehend the enormous significance and unavoidable requirements of building a socialist cultural power, adhere to a global and long-term vision, recognize the strategic importance of culture, strengthen the sense of mission and responsibility to promote cultural construction, and strive to realize the Chinese nation's cultural rejuvenation. As Shaanxi has unique and rich cultural resources, it is critical to explore and further revitalize these cultural resources as part of the province's overall economic and social development. The tourism competitiveness of smart tourism cities is evaluated using the BPNN model, and an empirical study is conducted in 10 smart tourism cities. The qualitative and quantitative index data are thoroughly investigated using the designed index system of tourism competitiveness of smart tourism cities. At the moment, audience segmentation for the dissemination of Shaanxi regional culture is insufficient, resulting in a loss of communication effect. Different audiences have varying levels of awareness of regional culture, and thus have varying levels of cultural recognition. Furthermore, cultural communication content, methods, channels, and skills all have an impact on the final communication effect, and these contents should be based on accurate audience research.

The article "Research on the Communication Strategy of History and Culture in Shaanxi Based on BP Neural Network Model" was published in 2022. Journal: Comput Intell Neurosci.

Although the BPNN model algorithm used in this paper is the most widely used algorithm in artificial neural networks, the samples chosen in this paper are somewhat fewer due to objective condition limitations, which reduces the accuracy and precision of BPNN model evaluation to some extent. It will be necessary to improve the sample data and the accuracy of data evaluation in future research.

## Figures and Tables

**Figure 1:** Cultural evaluation index system of famous historical cities.

**Figure 2:** Structural equation model.

**Figure 3:** BPNN structure.

**Figure 4:** Schematic of BPNN training error.

**Figure 5:** Comparison of Xi'an traffic mode sharing rate.

**Figure 6:** Comparison of traffic mode sharing rate in Hanzhong.

**Figure 7:** Comparison of traffic mode sharing rate in Baoji.

**Figure 8:** Comparison chart of expected output and training output.

**Figure 9:** Comparison of output results of test sample expected value and training value.

**Figure 10:** Ranking of evaluation results of tourism competitiveness of smart tourism cities.

## Data Availability

The data used to support the findings of this study are included within the article.
